The article "Propofol Inhibits Thyroid Cancer Cell Proliferation, Migration, and Invasion by Suppressing SHH and PI3K/AKT Signaling Pathways via the miR-141-3p/BRD4 Axis" was published in 2021. Journal: J Healthc Eng.

# Propofol Inhibits Thyroid Cancer Cell Proliferation, Migration, and Invasion by Suppressing SHH and PI3K/AKT Signaling Pathways via the miR-141-3p/BRD4 Axis

**DOI:** 10.1155/2021/2704753

**Published:** 2021-12-16

**Authors:** Heming Zhang, Mingtao Tan, Jing Zhang, Xiao Han, Yue Ma

**Affiliations:** ^1^Department of Anesthesia Surgery, Jinan Seventh People's Hospital, Jinan 250101, Shandong Province, China; ^2^Department of Anesthesiology, Zibo Central Hospital, Zibo 255036, Shandong Province, China; ^3^Department of Anesthesia Surgery, Zibo Central Hospital, Zibo 255020, Shandong Province, China; ^4^Department of Nuclear Medicine Radiotherapy, Zibo Central Hospital, Zibo 255036, Shandong Province, China; ^5^Department of Anesthesiology, Affiliated Hospital of Hebei University, Baoding 071000, Hebei Province, China

## Abstract

**Objective:**

This study explores the effect and mechanism of propofol for thyroid tumor.

**Methods:**

Culture human normal thyroid cells Nthy-ori 3-1 and thyroid cancer cell line TPC-1. TPC-1 cells were divided into the propofol group (treated with propofol), miR-141-3p group (transfected with the miR-141-3p mimic), negative control group (transfected with miR-NC), miR-141-3p + pcDNA-BRD4 group (transfected with the miR-141-3p mimic and pcDNA-BRD4), miR-141-3p + pcDNA group (transfected with the miR-141-3p mimic and pcDNA), siBRD4 group (transfected with siBRD4), and si-control group (transfected with si-control). The detection of miR-141-3p and BRD4 expression in cells was done by RT-qPCR, and the dual-luciferase reporter gene method and western blotting were used to verify the targeting relationship between miR-141-3p and BRD4. MTT method was used to test cell proliferation, transwell method was used to test cell migration and invasion, and western blotting was used to test SHH, GLI1, p-PI3K, and p-AKT protein expression.

**Results:**

Compared with Nthy-ori 3-1 cells, the expression of miR-141-3p in TPC-1 cells was markedly decreased. Propofol treatment and excessive expression of miR-141-3p could influence the phenotype of TPC-1 cells. BRD4 is one of the target genes of miR-141-3p, and its expression is negatively regulated by miR-141-3p. Overexpression of BRD4 can partially reverse the restraining effect of miR-141-3p on the TPC-1 cell phenotype. Both miR-141-3p and BRD4 can regulate the activity of SHH and PI3K/AKT signaling pathways.

**Conclusion:**

Propofol can inhibit the activity of SHH and PI3K/AKT pathways by targeting downregulating BRD4 through miR-141-3p, thereby inhibiting the phenotype of TPC-1 cells.

## 1. Instruction

Thyroid cancer, including papillary carcinoma, follicular cancer, undifferentiation carcinoma, and medullary carcinoma, is the most common malignant tumor of the thyroid. Papillary thyroid cancer (PTC), which is less malignant and has a better prognosis, is the most common [1]. The morbidity is related to locality, race, and sexual distinction. The incidence of women is higher, and the incidence is on the rise [2]. Data in 2018 showed that the number of women suffering from thyroid cancer in China accounted for 7.7% of the total cases [3].

The article "Propofol Inhibits Thyroid Cancer Cell Proliferation, Migration, and Invasion by Suppressing SHH and PI3K/AKT Signaling Pathways via the miR-141-3p/BRD4 Axis" was published in 2021. Journal: J Healthc Eng.

MicroRNAs (miRNAs) are a class of evolutionarily conserved, approximately 22-nucleotide long noncoding small RNAs. Their complementary binding with target mRNA can induce its degradation or prevent the translation of target mRNA to participate in the posttranscription regulation of target genes, which play an essential role in body development, homeostasis, and diseases [4]. miR-141-3p is a member of the miR-200 cluster, and its coding gene is located on chromosome 14. At present, low abundance of miR-14-3p is found in glioblastoma, pancreatic cancer, esophageal cancer, and other tumor tissues, while highly expressing miR-141-3p is found in mammary cancer and other tumors [5–7]. miR-141-3p regulates the growth of cancer cells and plays different roles in different tumor cells [8, 9].

Propofol is one of the most commonly used narcotics during cancer resection. Relevant studies have shown that propofol may suppress the invasion of human tumor cells [10, 11]. Zhang et al. showed that propofol can suppress the activity of cholangiocarcinoma cells and block the cell cycle to induce apoptosis [12]. At present, there are few studies on the effect of miR-141-3p in thyroid cancer. The effect of propofol on miR-141-3p expression in thyroid cancer cells has not been reported. Accordingly, our study intends to discuss the mechanism of propofol in the progression of thyroid cancer, so as to provide theoretical reference to the therapy of thyroid carcinoma.

## 2. Materials and Methods

### 2.1. Cell Culture and Propofol Treatment

Nthy-ori 3-1 and TPC-1 cells (from Shanghai Xuanya Biotechnology) were cultured in a 37°C incubator (from Thermo Fisher) containing 5% volume fraction of CO_2_. The medium is DMEM (from Life Technologies) involving 10% FBS (from Life Technologies), 10 mg/mL streptomycin, and 10k U/mL penicillin (from Sangon Biotech). TPC-1 cells in the logarithmic growth period were treated with propofol (from Novartis China) and cultured overnight.

### 2.2. Cell Transfection

TPC-1 cells in the logarithmic growth period were seeded and incubated in 6-well plates at the density of 3 × 10^3^ cells per well. When the cells' growth density reached about 50%, they were transfected according to the Lipofectamine 2000 transfection reagent manual. TPC-1 cells were transfected with miR-141-3p mimic, miR-NC, pcDNA-BRD4 + miR-141-3p mimic, pcDNA + miR-141-3p mimic, siBRD4, and si-control (from RiboBio).

The article "Propofol Inhibits Thyroid Cancer Cell Proliferation, Migration, and Invasion by Suppressing SHH and PI3K/AKT Signaling Pathways via the miR-141-3p/BRD4 Axis" was published in 2021. Journal: J Healthc Eng.

### 2.3. Cell Viability Assay

The cells were seeded in 96-well plates at the density of 1 × 10^5^ cells per well for 72 hours, and then 50 *μ*g MTT was added to each well. After shaking and mixing, the cells were cultured in a 37°C incubator including 5% volume fraction of CO_2_ for 4 hours. After incubation, the supernatant was removed, and 100 *μ*l DMSO (from Sigma-Aldrich) was added into every well and oscillated for 10 min to completely dissolve. The absorbance of each hole was determined at 490 nm by using the enzyme-labeled instrument (from Molecular Devices). Cell proliferation rate (%) = *A* (propofol)/*A* (control) × 100%.

### 2.4. Cell Migration Assay

The cells were digested with trypsin (from Gibco), the cell concentration was adjusted to about 2 × 10^5^/mL, and then they were inoculated in a transwell well (from Corning). 100 *μ*L of TPC-1 cell suspension was added to the upper well, and 500 *μ*L of the medium (containing 10% FBS) was added in the lower well. It was incubated for 24 hours, and the well was taken out and rinsed with PBS solution twice, then fixed with 4% paraformaldehyde for 15 minutes, and, finally, stained with crystal violet solution. After the transwell plate was dried, it was observed under an inverted microscope (from LASPEC), 5 visual fields were random choice for photographing, and the number of cells invading under the filter membrane in each visual field was counted.

### 2.5. Cell Invasion Assay

The cells were digested with trypsin, the cell concentration was adjusted to about 2 × 10^5^/mL, and then they were inoculated in a Matrigel-coated transwell well. 100 *μ*L of TPC-1 cell suspension was added to the upper well, and 500 *μ*L of the medium (containing 10% FBS) was added in the lower well. It was incubated for 24 hours, and the well was taken out and rinsed with PBS solution twice, then fixed with 4% paraformaldehyde for 15 minutes, and, finally, stained with crystal violet solution. After the transwell plate was dried, it was observed under an inverted microscope, 5 visual fields were random choice for photographing, and the number of cells invading under the filter membrane in each visual field was counted.

### 2.6. Real-Time Quantitative PCR (RT-qPCR)

The cells in the logarithmic growth phase were collected, total RNA was extracted from these cells with TRIzol test kits (from Thermo Fisher), and cDNA was synthesized according to the reverse transcription kit (from Invitrogen). cDNA was used as the template to perform RT-qPCR test to sense the abundance of miR-141-3p and BRD4 in these cells. The relative abundance was calculated by the 2^−ΔΔCt^ method. The internal reference is U6. The sequence of primers used in this experiment (from Sangon Biotech) is shown in Table 1.

The article "Propofol Inhibits Thyroid Cancer Cell Proliferation, Migration, and Invasion by Suppressing SHH and PI3K/AKT Signaling Pathways via the miR-141-3p/BRD4 Axis" was published in 2021. Journal: J Healthc Eng.

### 2.7. Dual-Luciferase Reporter Gene Method

The bioinformatics online database TargetScan was used to forecast the targeted gene of miR-141-3p. The results showed that there was a targeted binding site between the 3′-UTR of BRD4 and miR-141-3p, indicating that BRD4 is probably the targeting gene of miR-141-3p. The luciferase recombinant vectors containing wild-type BRD4 3′-UTR (BRD4-Wt) and mutant BRD4 3′-UTR (BRD4-Mut) were amplified and constructed, respectively. The BRD4-Wt or BRD4-Mut recombinant vectors were cotransfected with miR-141-3p mimic and miR-con into TPC-1 cells, respectively. After 48 hours, the luciferase activity was measured using the dual-luciferase activity detection kit (from Promega) to calculate the relative fluorescence activity of cells.

### 2.8. Western Blotting

Each group of cells was taken and added cell lysate (from Beyotime Biotechnology) and then incubated on ice for 30 minutes. The protein in the cells was collected, and the total protein was quantified with the BCA protein detection kit (from Beyotime Biotechnology). 50 *μ*g protein sample was taken, and the protein was separated with 12% sodium lauryl sulfate-polyacrylamide gel, transferred to the nitrocellulose membrane (from Sigma), and blocked for 1 hour. Protein primary antibody (from Abcam) was added and incubated overnight at 4°C. Secondary antibodies (from Abcam) were added at room temperature on the next day, incubated for 1 hour, and placed in the gel imaging system for exposure, and Quantity One software was used to analyze the gray value of protein bands.

### 2.9. Statistical Analysis

Statistical software SPSS 17.0 and GraphPad Prism 8.0.2 were used for statistical analysis of experimental data. Statistical data were expressed as mean ± standard deviation (*x* ± *s*), *t*-test. The count data were described by the utilization rate (%). *P* < 0.05 represents that the difference had a statistical significance.

## 3. Results

### 3.1. Propofol Suppresses Proliferation, Migration, and Invasion of Thyroid Cancer Cells

In this experiment, MTT method and transwell method were used to test the influences of propofol on the phenotype of thyroid cancer cells. From results compared with the control group (0 *μ*g/L), the activity of TPC-1 cells in the propofol group was significantly decreased (Figure 1), and their migration and invasion were also significantly inhibited (Figure 2).

### 3.2. miR-141-3p Suppresses Proliferation, Migration, and Invasion of Thyroid Cancer Cells

The abundance of miR-141-3p in thyroid cancer cells was detected by RT-qPCR. We found that the abundance of miR-141-3p in TPC-1 cells was significantly decreased than that in Nthy-ori 3-1 cells (*P* < 0.001, Figure 3(a)). In order to study the influence of miR-141-3p on the activity of TPC-1 cells, we used miR-141-3p mimic to induce the expression of miR-141-3p in TPC-1 cells. As shown in Figure 3(b) (*P* < 0.001), the abundance of miR-141-3p in TPC-1 cells transfected with miR-141-3p mimic was obviously superior than that in the negative control, indicating that the cells' excessive expression miR-141-3p had been successfully established. MTT and transwell results showed that overexpression of miR-141-3p obviously inhibited the phenotype of TPC-1 cells (all *P* < 0.05, Figures 3(c)–3(e)).

The article "Propofol Inhibits Thyroid Cancer Cell Proliferation, Migration, and Invasion by Suppressing SHH and PI3K/AKT Signaling Pathways via the miR-141-3p/BRD4 Axis" was published in 2021. Journal: J Healthc Eng.

### 3.3. miR-141-3p Expression Is Promoted by Propofol

The expression of miR-141-3p in TPC-1 cells treated with propofol for 24 hours was detected by RT-qPCR, and we found that the expression of miR-141-3p in TPC-1 cells was obviously increased (*P* < 0.001, Figure 4).

### 3.4. BRD4 Is the Targeting Gene of miR-141-3p

TargetScan prediction result displayed that there was a specific binding site between miR-141-3p and BRD4 3′-UTR (Figure 5(a)). After wild-type BRD4 luciferase expression vector WT-BRD4 was cotransfected with miR-141-3p mimics or miR-con into TPC-1 cells, respectively, the luciferase activities of TPC-1 cells in the miR-141-3p group were obviously decreased than those in miR-con (*P* < 0.001). However, after cotransfection of mutant BRD4 luciferase expression vector MUT-BRD4 with miR-141-3p mimic or miR-con on TPC-1 cells, the difference was not statistically significant in luciferase activity between the miR-141-3p group and miR-con (*P* > 0.05) (Figure 5(b)).

### 3.5. Propofol Suppresses the SHH and PI3K/AKT Pathways

According to the analysis of western blotting results, the protein abundance of SHH, GLI1, p-PI3K, and p-AKT was inhibited after propofol treatment for 24 hours (*P* < 0.01, Figure 6(a)).

### 3.6. SHH  and PI3K/AKT Pathways Are Regulated by miR-141-3p Expression

As shown in Figure 6(b), the protein abundance of SHH, GLI1, p-PI3K, and p-AKT in TPC-1 cells after overexpression of miR-141-3p was lower than that in the untransfected and transfected miR-NC groups (*P* < 0.01).

### 3.7. SHH and PI3K/AKT Pathways Are Regulated by BRD4 Expression

As shown in Figure 6(c), compared with the cells in the untransfected and transfected si-control groups, the protein abundance of SHH, GLI1, p-PI3K, and p-AKT in TPC-1 cells decreased after BRD4 was silenced (*P* < 0.001).

The article "Propofol Inhibits Thyroid Cancer Cell Proliferation, Migration, and Invasion by Suppressing SHH and PI3K/AKT Signaling Pathways via the miR-141-3p/BRD4 Axis" was published in 2021. Journal: J Healthc Eng.

### 3.8. BRD4 Overexpression Partially Reversed the Influences of miR-141-3p on TPC-1 Cell Activity

As shown in Figure 7, compared with the miR-141-3p + pcDNA group, the phenotype of TPC-1 cells in the miR-141-3p + pcDNA-BRD4 group was significantly promoted (*P* < 0.05).

## 4. Discussion

Propofol is one of the frequently used narcotics for cancer resection. Since Mammoto et al. first proposed in 2002 that clinical related concentrations of propofol could inhibit the invasion of human cancer cells (cervical cancer HeLa cells, fibrosarcoma HT1080 cells, osteosarcoma HOS cells, and melanoma RPMI-7951 cells) [13], its effect on tumor cells and its mechanism have become a rapidly developing topic and gradually attracted extensive attention. Related studies have shown that propofol can inhibit the invasion and metastasis of esophageal squamous cell carcinoma cells by downregulating the expression of SOX4 [14]. In addition, propofol can also inhibit invasion and angiogenesis and induce apoptosis of esophageal cancer EC-1 cells in vitro by regulating the expression of S100A4 [15]. Chen et al. showed that propofol could inhibit the migration of pancreatic cancer cells by inhibiting NMDA receptors [16]. In addition, propofol can also inhibit the proliferation, invasion, and metastasis of pancreatic cancer cells and induce apoptosis of tumor cells by upregulating the expression of miR-133a and miR-21 [17, 18]. Li et al. found that propofol can inhibit the phenotype of PTC cells by inhibiting the activation of the NF-*κ*B pathway and Wnt/*β*-catenin [19]. This is consistent with the results of this experiment; we found that the phenotype of TPC-1 cells treated with propofol was significantly inhibited, suggesting that propofol had a certain restraining effect on the malignant behavior of thyroid tumor cells.

Relevant research studies have already shown that the antitumor influence of propofol perhaps is closely in connection with miRNA it regulates. For example, propofol can inhibit the proliferation of mammary cancer MCF-7 cells by downregulating the expression of miR-21 [20] and can also inhibit the activity of melanoma cells by adjusting miR-137 and FGF9 [21]. miRNAs play important roles in development, cell differentiation, hematopoietic function, cell apoptosis, growth, and immune system. Many human diseases including cancer, autoimmune diseases, and chronic diseases are related to the abnormal regulation of miRNA. Dong et al. found that miR-141 was downregulated in thyroid tumor tissue [22], which equates with our study. We found that propofol could increase the abundance of miR-141-3p in TPC-1 cells. To verify the role of miR-141-3p in thyroid cancer, we overexpressed miR-141-3p in thyroid cancer cells. The results showed that overexpression of miR-141-3p inhibited the phenotype of TPC-1 cells. It is speculated that miR-141-3p may play an important role in the antithyroid cancer mechanism of propofol.

The article "Propofol Inhibits Thyroid Cancer Cell Proliferation, Migration, and Invasion by Suppressing SHH and PI3K/AKT Signaling Pathways via the miR-141-3p/BRD4 Axis" was published in 2021. Journal: J Healthc Eng.

BRD4 is one of the members of the bromodomain and extraterminal domain (BET) family, which is an essential epigenetic regulator of gene transcription and cancer development. As one of them, BRD4 can regulate various characteristics of cancer cells by adjustment of the expression and activity of cancer promoters, including drug resistance, apoptosis, cell transformation, proliferation, and invasion [23]. BRD4 is overexpressed in a variety of parenchymatous tumors, including pancreatic cancer, mammary cancer, and colorectal cancer, and its expression inhibition can hinder the invasion and proliferation of these tumor cells [24, 25]. In this study, we predicted and proved that BRD4 is a targeted gene of miR-141-3p by bioinformatics, and overexpression of BRD4 can partially reverse the inhibitory effect of miR-141-3p on the phenotype of thyroid cancer cells. It is speculated that miR-141-3p may inhibit the malignant behavior of thyroid cancer cells by regulating the abundance of BRD4.

SHH and PI3K/AKT are both pathways that play important roles in cancer progression. SHH is involved in tumor metastasis in basal cell carcinoma, ovarian cancer, cervical cancer, breast cancer, gastric cancer, and pancreatic cancer and is related to drug resistance and survival of cancer [26–31]. Among the disordered signaling pathways, PI3K/AKT pathway is the most frequently changed signaling pathway. AKT is a Ser/Thr protein kinase and an important node in the PI3K signaling pathway. It has three different subtypes, AKT1, AKT2, and AKT3, which are closely related to the development of human cancer [32, 33]. Previous research studies have shown that BRD4 can promote the phenotype of thyroid cancer cells through the SHH pathway. In addition, downregulation of BRD4 in GBC cells can induce apoptosis through the PI3K/AKT pathway. In the current study, we obtained the conclusion that propofol treatment, overexpression of miR-141-3p, and silencing BRD4 can downregulate the abundance of SHH and PI3K/AKT pathway-related proteins SHH, GLI1, p-PI3K, and p-AKT and inhibit SHH and PI3K/AKT signal pathways' activation.

In summary, our study confirmed the inhibition of propofol for the malignant behavior of thyroid tumor. Its antitumor effect may be achieved by regulating miR-141-3p to target BRD4 affecting the activity of SHH and PI3K/AKT signaling pathways. However, there are many related factors that regulate the behavior of thyroid cancer cells; this study still has certain limitations. The specific mechanism of propofol's inhibitory effect on thyroid cancer cells needs to be further studied.

The article "Propofol Inhibits Thyroid Cancer Cell Proliferation, Migration, and Invasion by Suppressing SHH and PI3K/AKT Signaling Pathways via the miR-141-3p/BRD4 Axis" was published in 2021. Journal: J Healthc Eng.

## Figures and Tables

**Figure 1:** Effect of propofol on proliferation of TPC-1 cells (^*∗∗∗*^*P* < 0.001).

**Figure 2:** Effect of propofol on migration and invasion of TPC-1 cells. Propofol can inhibit the migration (a) and invasion (b) of TPC-1 cells (^*∗*^*P* < 0.05).

**Figure 3:** The abundance of miR-141-3p in TPC-1 cells and its influence on the biological behavior of cancer cells. (a) Compared with Nthy-ori 3-1 cells, the expression of miR-141-3p in TPC-1 cells was significantly decreased (^*∗∗∗*^*P* < 0.001). (b) The abundance of miR-141-3p was successfully increased in TPC-1 cells by using miR-141-3p mimics (^*∗∗∗*^*P* < 0.001). (c–e) Overexpression of miR-141-3p significantly inhibited the phenotype of TPC-1 cells (^*∗*^*P* < 0.05 and ^*∗∗∗*^*P* < 0.001).

**Figure 4:** Propofol promotes miR-141-3p expression in TPC-1 cells (^*∗∗∗*^*P* < 0.001).

**Figure 5:** BRD4 is a targeting gene of miR-141-3p in TPC-1 cells. (a) A complement sequence of miR-141-3p is found in the 3′-UTR of BRD4. (b) Dual-luciferase reporter gene analysis proved the interaction of miR-141-3p and BRD4 (^*∗∗∗*^*P* < 0.001).

**Figure 6:** Influences of propofol (a), miR-141-3p (b), and BRD4 (c) on the expressions of key proteins related to SHH and PI3K/AKT pathways (^*∗∗*^*P* < 0.01 and ^*∗∗∗*^*P* < 0.001).

**Figure 7:** Cell proliferation (a), migration (b), and invasion (c) are all promoted by overexpression of BRD4 in TPC-1 cells (^*∗*^*P* < 0.05).

**Table 1:** Primer sequences of RT-qPCR.

Gene	Sequence
miR-141-3p	F: 5′-GCGGCGGTAACACTGTCTGG-3′
	R: 5′-AACGCTTCACGAATTTGCGT-3′

BRD4	F: 5′-GCACAATCAAGTCTAAACTGGAG-3′
	R: 5′-TCATGGTCAGGAGGGTTGTAC-3′

U6	F: 5′-GCTTCGGCAGCACATATACTAAAAT-3′
	R: 5′-CGCTTCACGAATTTGCGTGTCAT-3′

## Data Availability

The data used to support the findings of this study are available from the corresponding author upon reasonable request.
